# Theory-Based Failure Modes and Effect Analysis for Medication Errors

**DOI:** 10.1155/2021/5533208

**Published:** 2021-03-31

**Authors:** Saeid Jafarzadeh Ghoushchi, Shadi Dorosti, Mohd Nizam Ab Rahman, Marzieh Khakifirooz, Mahdi Fathi

**Affiliations:** ^1^Faculty of Industrial Engineering, Urmia University of Technology, Urmia, Iran; ^2^Department of Mechanical and Manufacturing Engineering, Faculty of Engineering and Built Environment, Universiti Kebangsaan Malaysia, Bangi, Selangor, Malaysia; ^3^Department of Industrial Engineering, Tecnologico de Monterrey, Monterrey,NL, Mexico; ^4^Department of Information Technology & Decision Sciences, G. Brint Ryan College of Business, University of North Texas, Denton, TX, USA

## Abstract

Medication Errors (MEs) are still significant challenges, especially in nonautomated health systems. Qualitative studies are mostly used to identify the parameters involved in MEs. Failing to provide accurate information in expert-based decisions can provoke unrealistic results and inappropriate corrective actions eventually. However, mostly, some levels of uncertainty accompany the decisions in real practice. This study tries to present a hybrid decision-making approach to assigning different weights to risk factors and considering the uncertainty in the ranking process in the Failure Modes and Effect Analysis (FMEA) technique. Initially, significant MEs are identified by three groups of qualified experts (doctors, nurses, and pharmacists). Afterward, for assigning weights to the risk factors, *Z*-number couples with the Stepwise Weight Assessment Ratio Analysis (SWARA) method, named *Z*-SWARA, to add reliability concept in the decision-making process. Finally, the identified MEs are ranked through the developed Weighted Aggregated Sum Product Assessment (WASPAS) method, namely, *Z*-WASPAS. To demonstrate the applicability of the proposed approach, the ranking results compare with typical methods, such as fuzzy-WASPAS and FMEA. The findings of the present study highlight improper medication administration as the main failure mode, which can result in a fatality or patient injury. Moreover, the utilization of multiple-criteria decision-making methods in combination with *Z*-number can be a useful tool in the healthcare management field since it can address the problems by considering reliability and uncertainty simultaneously.

## 1. Introduction

Medication Errors (MEs) are the most common medical error that can disproportionately affect patients [1]. According to the available statistics, MEs affect approximately 1.5 million people each year [2]. MEs can occur throughout the medication-use system, such as prescribing medication, entering information into a system when medication is being prepared or dispensed, or when medication is given to or taken by a patient. Indeed, MEs are avoidable occurrences that may typically cause improper medication usage or patient damage. Hence, to prevent patients' injury or fatality, health centers endeavor to make practical measurements and develop various systems for MEs minimization [3].

One of the trends for reducing MEs is establishing advanced medication systems which are adopted in some countries, including the United States [4], Malaysia [5], New Zealand [6], and China [7]. However, improving systems depends on monitoring all steps of medical services and true recognition of failure modes to eliminate the problem [8]. Failure Modes and Effect Analysis (FMEA) is a systematic tool to identify the potential failures, causes and effects of failures, and provide preventive actions [9, 10]. Therefore, it is an appropriate approach to use in the health-care field [11–13] and recognize possible failure modes in the MEs process [14, 15]. Based on the FMEA method, the risk priorities of the failure modes are specified through the Risk Priority Number (RPN) value. The RPN is the result of the occurrence, severity, and detection of potential failure modes multiplication [16, 17]. However, RPN scores have been criticized for some deficiencies, including uncertainty in team-based decision making, the shortage of full ranking for risks, and assumption of the equal importance of risk factors and not considering uncertainty concept [18–20]. Notably, to deal with the uncertainty in solving risk analysis problems, there are various useful theories including R-Number, G-number, and evidence theory [21–23]. Therefore, to address the shortcomings of RPN, it is necessary to develop a novel prioritization approach for prioritizing the identified MEs using Multiple-Criteria Decision-Making (MCDM) methods [24, 25]. In the meantime, the combination of the FMEA technique with the data envelopment analysis [12], best-worst method [19], MOORA [13], VIKOR [17], gray relational projection [21], and TOPSIS [24] can be mentioned.

Recently, researchers attend to apply MCDM methods in complicated decision-making processes, including healthcare sectors [26, 27]. For instance, Mardani et al. [26] concluded MCDM methods as effective techniques in different sections of hospitals and health centers to facilitate complex decisions making processes, assess various health centers and health services, and resolve uncertainty in different levels of decisions in healthcare centers. Hsieh et al. [27], for the first time, applied MCDM methods for reducing MEs. In their study, the Analytic Hierarchy Process (AHP) and technique for order of preference by similarity to ideal solution (TOPSIS) are applied to evaluate the crucial human error factors that are associated with MEs events. Besides, in the past years, researchers suggested various strategies to reduce MEs, for instance, utilizing lean six sigma method [28], simulation-based learning [29, 30], logistic regression [31], and carrying out qualitative studies [32].

The main contribution of this study is to provide an integrated approach to cover the deficiencies of traditional RPN score. Besides, the cost and time factors are added to RPN scoring because they are playing significant roles in MEs [33, 34]. In other words, MEs can be costly for both hospitals and patients and waste the time of proper treatment. In this paper, initially, ten main failure modes that induce the MEs are introduced by experts based on the FMEA method. Thereafter, with the aims of assigning weight to the quintuple factors of RPN, a combination of the *Z*-number and Stepwise Weight Assessment Ratio Analysis (SWARA) method, named *Z*-SWARA, is utilized. The *Z*-number theory is applied for considering the uncertainty and reliability simultaneously in expressing the values of RPN factors for each failure mode. In this way, the deficiencies of conventional FMEA are addressed by assigning different weights to RPN factors based on their importance. The SWARA method has the advantage of a more logical calculation of weights and relative importance of criteria. The ability to estimate experts' opinions about the importance ratio of the criteria in the process of their weight determination is the main element of this method [35]. Moreover, this method helps coordinate and gather data from experts. Furthermore, the SWARA method is uncomplicated, and experts can easily work together. The main advantage of this method in decision making is that in some problems priorities are defined based on policies of companies or countries and there are not any needs for evaluation to rank criteria [36]. In the third phase, the extended version of Weighted Aggregated Sum Product Assessment (WASPAS) using *Z*-number theory (*Z*-WASPAS) is applied for ranking ten failure modes, considering reliability in addition to the uncertainty using the *Z*-number theory, in comparison with fuzzy theory. The *Z*-numbers theory, like the *D*-numbers theory extended based on the Dempster–Shafer theory, represents an approach for intending uncertainty and imprecision in expert decisions [37]. In comparison with *D*-numbers theory, *Z*-numbers consider the fuzzy information and reliability of this information simultaneously. This theory is an effective tool to express the uncertainty in expert preferences, which is based on the reliability of choosing the appropriate criterion value. The main advantage of the WASPAS method is its high degree of reliability. Integration of rough numbers and the WASPAS method with advantages of both concepts presents very important support in decision-making in everyday conflicting situations [38].

The remainder of this paper is organized as follows: Section 2 introduces the fundamental theorem of *Z*-number followed by SWARA and WASPAS methods and transformation rules to *Z*-WASPAS and *Z*-SWARA. In Section 3, the research framework and ten main failure modes resulting in MEs are presented. In Section 4, the validation results of the proposed method in comparison with traditional methods are indicated. The suggested actions to remove or reduce failure modes and future research directions are compromised in Section 5.

## 2. Methodology

To explain the proposed approach, first, *Z*-number is introduced as a reliability increment method, along with the preliminary definitions and mathematical equations. Afterward, transformation rules are discussed in detail for both *Z*-SWARA and *Z*-WASPAS methods for ranking failure modes. In this study, the terms “failure mode” and “alternative” and “criteria” and “risk factors” are used interchangeably. Moreover, for simplicity, the fuzzy number term is used for the specific Triangular Fuzzy Number (TFN).

### 2.1. Terminologies and Notations

The mathematical terminologies and notations used in this study are as follows:

- *Y*: universal set
- *y*: membership of *Y*
- $\tilde{G}$: a fuzzy set
- $\mu_{\tilde{G}}\left(y\right)$: membership function of dependency *y* ∈ *Y* in $\tilde{G}$ set
- (*a*, *b*, *c*): lower, medium, and upper bounds of TFN
- *R*(*Y*): fuzzy restriction in *Y* domain
- $Z=\left(\tilde{F},\tilde{L}\right)$: a *Z*-number with the first component $\tilde{F}$ and second component $\tilde{L}$
- $\tilde{F}$: restriction component of *Z*-number with membership function of $\mu_{\tilde{F}}\left(y\right)$
- $\tilde{L}$: reliability of restriction component in the *Z*-number with membership function of $\mu_{\tilde{L}}\left(y\right)$
- *i*: failure mode/alternative index
- *j*: risk factor/criteria index
- *m*: number of alternatives (*m*=1,…, *i*)
- *n*: number of criteria (*n*=1,…, *j*)
- *α*: crisp value
- ${\tilde{Z}}_{j}^{\prime }$: converted form of weighted *Z*-number to TFN for *j*-th criteria
- ${\tilde{q}}_{j}$: fuzzy weight coefficient for *j*-th criteria
- ${\tilde{w}}_{j}$: fuzzy relative weight for *j*-th criteria
- *K*_*i*_: the utility function for *i*-th alternative
- *H*: decision-making matrix with the *Z*-number elements
- *h*_*ij*_: elements of matrix *H*
- *H*: converted decision-making matrix with the TFN elements
- ${\tilde{\bar{h}}}_{ij}$: elements of matrix *H*
- ${\hat{h}}_{ij}$: normalized form of the elements of *H* decision-making matrix
- ${\tilde{Q}}_{i}$: weighted sum for *i*-th alternative
- ${\tilde{P}}_{i}$: weighted product for *i*-th alternative

### 2.2. Preliminary Definitions and Concepts

In this section, preliminary concepts required to develop the proposed approach of this study are presented.

*Fuzzy Set*. A fuzzy set is a membership function that shows a degree of membership in [0,1] interval. In (1), a fuzzy set like $\tilde{G}$ defines *y*, the membership value, in *Y* reference set [39]:

(1) $$\begin{array}{c} \tilde{G}=\left\{y|\mu_{\tilde{G}}:\;Y\;⟶\;\left[0,1\right],\;\;y\in Y\right\}, \end{array}$$

where $\mu_{\tilde{G}}\left(y\right)$ represents the degree of belonging of *y* ∈ *Y* in $\tilde{G}$ set.

*TFN*. The triplet (*a*, *b*, *c*) set is known as TFN. The membership function of a TFN like $\tilde{G}=\left(a,b,c\right)$ is [40]

(2) $$\begin{array}{c} \mu_{\tilde{G}}\left(y\right)=\left\{\begin{array}{cc} \frac{y-a}{b-a}, & a\leq y\leq b,\\ 1, & y=b,\\ \frac{c-y}{c-b}, & b\leq y\leq c,\\ o & \text{otherwise}. \end{array}\right) \end{array}$$

In this study, the TFN form of fuzzy numbers is considered.

*Fuzzy Restriction*. A fuzzy restriction is visualized as an elastic constraint on the values that are assigned to a variable. A restriction may be viewed as a generalized constraint. Suppose $\tilde{F}$ is a fuzzy set; the restriction *R*(*Y*) is as a probabilistic constraint such that [41]

(3) $$\begin{array}{c} R\left(Y\right):Y\text{ is }\tilde{F}, \end{array}$$

where $\tilde{F}$ is playing the role of the possible distribution of *Y*.

The statement in equation (3) can be interpreted as follows:

(4) $$\begin{array}{c} R\left(Y\right):Y\text{ is }\tilde{F}\;⟶\text{poss}\left(Y=y\right)=\mu_{\tilde{F}}\left(y\right), \end{array}$$

where $\mu_{\tilde{F}}$ is a membership function of *F* and *y* is a generic value of *Y*. $\mu_{\tilde{F}}$ can be constrained how $\tilde{F}$ is associated with *R*(*Y*).

*Z*-*Number Theory*. A *Z*-number is an ordered pair of $\left(\tilde{F},\tilde{L}\right)$, where $\tilde{F}$ and $\tilde{L}$ are assumed to be TFN. A *Z*-number associated with a real-valued uncertain variable **Y**, where $\tilde{F}$, as a first component, is a fuzzy subset from **Y** domain, and $\tilde{L}$ is a fuzzy subset from a unite interval [0, 1] [42]. A *Z*-number can provide information about an uncertain variable, where $\tilde{F}$ is the restriction and $\tilde{L}$ represents an idea of certainty or reliability. A collection of *Z*-valuations is referred to as *Z*-information. It should be noted that much of everyday reasoning and decision-making is based, in effect, on *Z*-information. According to the fuzzy restriction in equation (2), suppose that *Y* is a random variable; its probability distribution of *Y* illustrates the probabilistic restriction on *Y*. The probabilistic restriction is

(5) $$\begin{array}{c} R\left(Y\right):Y\text{ is }p, \end{array}$$

and based on equation (5), the probability density function of *Y* is explained in the following equation:

(6) $$\begin{array}{c} R\left(Y\right):Y\text{ is }p⟶\text{prob}\left(u\leq Y\leq u+\text{d}u\right)=p\left(u\right)\text{d}u, \end{array}$$

where *p* is the probability density function of *Y* and d*u* represents deferential of *u*.

To convert *Z*-number to TFN, assume first that *Z*=[(*a*_1_, *b*_1_, *c*_1_), (*a*_2_, *b*_2_, *c*_2_)]; the first part (*a*_1_, *b*_1_, *c*_1_) plays the role of restriction and the second part (*a*_2_, *b*_2_, *c*_2_) represents reliability [43]. Initially, the second part (reliability) converts into a crisp number, *α*, as follows:

(7) $$\begin{array}{c} \alpha =\frac{\int y\;\mu_{\tilde{L}}\left(y\right)\text{d}y}{\int \mu_{\tilde{L}}\left(y\right)\text{d}y}, \end{array}$$

where $\mu_{\tilde{L}}\left(y\right)$ is as defined in equation (2).

Then, *α* as the weight of the second part (reliability) added to the first part (restriction), and the TFN form of weighted *Z*-number is obtainable through the following equation:

(8) $$\begin{array}{c} {\tilde{Z}}^{\prime }=\left(\sqrt{\alpha }*a_{1},\sqrt{\alpha }*b_{1},\sqrt{\alpha }*c_{1}\right). \end{array}$$

### 2.3. *Z*-SWARA Method

The fuzzy Stepwise Weight Assessment Ratio Analysis (fuzzy SWARA) is a multiple-attribute decision-making method [35] for calculating the weight of criteria and subcriteria [44] in a fuzzy environment. The fuzzy SWARA acts the same as the SWARA method [35], but the ambiguity in decision-making or incomplete information leads to the extension of the SWARA method to fuzzy SWARA. In the fuzzy SWARA method, experts play a significant role in assigning the weight of the criteria; therefore, the information accumulates based on experts' opinions [45–49]. In this study, the fuzzy SWARA method extended to the *Z*-SWARA method, and the reliability factor is added to enhance the certainty in the final results. The steps of the *Z*-SWARA method are as follows:

Step 1. Initially, the experts sort criteria, from the most important to less important in descending order, based on self-identification.
Step 2. Based on the initial opinion, experts need to assign linguistic variables to the relative importance of criteria *j* in relation to the previous *j* − 1 criteria. Thereafter, experts set the value of the first component (${\tilde{F}}_{j}$), according to Table 1 [40], and the reliability component $\left({\tilde{L}}_{j}\right)$ is assigned through Table 2 [43]. The result forms a *Z*-number for each criterion.
Step 3. To convert the *Z*-number as a result in Step 2 to a TFN, firstly, according to equation (6), the second part (reliability) converts into a crisp number, and the weight is added to the first part based on equation (7).
As a numerical example, suppose that for the *j*-th criteria, the relative importance in the form of linguistic variables is (VLI, *M*). By replacing the corresponding TFN values of VLI and *M* from Tables 3 and 4, respectively, the *Z*-number forms as [((2/7), (1/3), (2/5)), (0.35, 0.5, 0.75)]. The crisp value is *α*=0.53, and the TFN form of *Z*-number according to equation (7) is (0.21, 0.24, 0.29). Other transformations of *Z*-number to TFN are presented in Table 5.
Step 4. Based on the results of Step 3, coefficient ${\tilde{q}}_{j}$ as a fuzzy weight coefficient is defined as follows:
  (9) $$\begin{array}{c} {\tilde{q}}_{j}=\frac{{\tilde{q}}_{j-1}}{{\tilde{Z}}_{j}^{\prime }}, \end{array}$$
 where ${\tilde{q}}_{j}$ is TFN and ${\tilde{q}}_{1}=\left(1,1,1\right)$.
Step 5. Finally, considering *n* evaluation criteria, the relative weights of the *j*-th evaluation criteria are determined as follows:
  (10) $$\begin{array}{c} {\tilde{w}}_{j}=\frac{{\tilde{q}}_{j}}{\sum_{j=1}^{n}{\tilde{q}}_{j}}, \end{array}$$
 where ${\tilde{w}}_{j}$ is a TFN.

### 2.4. *Z*-WASPAS Method

The fuzzy-WASPAS is a multivariable decision-making method [50], which, such as the WASPAS method [51, 52], is usually used in highly sensitive cases by considering the certainty of the system [51] (for instance, see the example of reservoir flood control management in [53] and see the example of reservoir flood control management in [54]). The fuzzy-WASPAS method is a unique combination of two well-known MCDM approaches, the Weighted Sum Model (WSM) and Weighted Product Model (WPM). In the fuzzy-WASPAS method, the beneficial (e.g., profit, efficiency) or non-beneficial (e.g., cost) aspect of each risk factor must be determined based on experts' opinions. For the beneficial aspects higher values are always desirable, and for non-beneficial smaller values are always preferable. In this study, only beneficial aspects of criteria are considered, and the final output of fuzzy-WASPAS presents as a utility function (*K*_*i*_) that can help to rank alternatives. The new extended *Z*-number of fuzzy-WASPAS, namely, *Z*-WASPAS, is used for ranking failure modes. The steps of the *Z*-WASPAS method are as follows:

(i) *Step 1*. First, experts determine a linguistic variable for each element, and then the corresponding values of each linguistic variable are assigned to each element to make decision matrix *H*. Consider a *Z*-number like $Z=\left({\tilde{F}}_{ij},{\tilde{L}}_{ij}\right)$, linguistic value for ${\tilde{F}}_{ij}$ is selected using Table 3 [50], and similar to *Z*-SAWARA method, ${\tilde{L}}_{ij}$ can get the linguistic values from Table 4. Therefore, the decision-making matrix *H* with *Z*-number elements is determined as follows:
  (11) $$\begin{array}{c} H=\left[\begin{array}{ccc} h_{11} & \ldots & h_{1n}\\ \ldots & \ldots & \ldots \\ h_{m1} & \ldots & h_{mn} \end{array}\right], \end{array}$$
where *h*_*ij*_=[(*a*_*ij*_^*f*^, *b*_*ij*_^*f*^, *c*_*ij*_^*f*^), (*a*_*ij*_^*l*^, *b*_*ij*_^*l*^, *c*_*ij*_^*l*^)], *i*=1,…, *m*, *j*=1,…, *n*, *m* indicates the number of alternatives, and *n* shows the number of criteria.
(ii) *Step 2*. The decision matrix *H* with *Z*-number elements converts to TFN $\left({\tilde{Z}}^{\prime }\right)$. The transformed decision-making matrix *H* is as follows:
  (12) $$\begin{array}{c} \tilde{\bar{H}}=\left[\begin{array}{ccc} {\tilde{\bar{h}}}_{11} & \ldots & {\tilde{\bar{h}}}_{1n}\\ \ldots & \ldots & \ldots \\ {\tilde{\bar{h}}}_{m1} & \ldots & {\tilde{\bar{h}}}_{mn} \end{array}\right], \end{array}$$
where ${\tilde{\bar{h}}}_{ij}$ is a TFN in the form of ${\tilde{Z}}^{\prime }$, *i*=1,…, *m*, *j*=1,…, *n*, *m* indicates the number of alternatives, and *n* shows the number of criteria.
 As a numerical example, suppose that for the *i*th alternative and the *j*th criteria, the importance, ${\tilde{F}}_{ij}$, is determined “medium poor” (MP) and the reliability, ${\tilde{L}}_{ij}$, is selected “weak” (*W*) by the expert; consequently, the *Z*-number and the crisp value are [(2,3.5, 5), (0.20, 0.35, 0.50)], and *α*=0.35, respectively. Therefore, the transformed form of *Z*-number to a TFN $\left({\tilde{Z}}^{\prime }\right)$ is (1.18, 2.08, 2.96). Other transformations of *Z*-number to TFN $\left({\tilde{Z}}^{\prime }\right)$ are presented in Table 4.
(iii) *Step 3*. Normalize $\tilde{\bar{H}}$ matrix considering beneficial and nonbeneficial elements, using
  (13) $$\begin{array}{c} {\hat{h}}_{ij}=\left\{\begin{array}{cc} \frac{{\tilde{\bar{h}}}_{ij}}{\underset{i}{\max}\;{\tilde{\bar{h}}}_{ij}}, & \text{for }j\text{beneficial,}\\ \frac{\underset{i}{\min}{\tilde{\bar{h}}}_{ij}}{{\tilde{\bar{h}}}_{ij}}, & \text{for }i\text{nonbeneficial}. \end{array}\right) \end{array}$$
(iv) *Step 4*. Determine the weighted normalized fuzzy decision-making matrix of ${\hat{h}}_{ij}$ for the WSM ($\tilde{Q}$ TFN) and WPM ($\tilde{P}$ TFN) as follows:
  (14) $$\begin{array}{c} {\tilde{Q}}_{i}=\overset{n}{\underset{j=1}{\sum }}{\hat{h}}_{ij}{\tilde{w}}_{j}\\ {\tilde{P}}_{i}=\overset{n}{\underset{j=1}{\prod }}{\hat{h}}_{ij}^{{\tilde{w}}_{j}}. \end{array}$$
 To facilitate defuzzification of the performance measurement, center-of-area of each TFN is considered for decision making as follows [49]:
  (15) $$\begin{array}{c} {\bar{Q}}_{i}=\frac{1}{3}\left(a_{i}^{Q}+b_{i}^{Q_{i}}+c_{i}^{Q}\right),\\ {\bar{P}}_{i}=\frac{1}{3}\left(a_{i}^{P}+b_{i}^{P}+P_{i}^{c}\right). \end{array}$$
(v) *Step 5*. Calculate the value of failure modes and rank them using utility function *K*_*i*_ for *i*th alternative as follows:
  (16) $$\begin{array}{c} K_{i}=\lambda \sum_{j=1}^{m}{\bar{Q}}_{i}+\left(1-\lambda \right)\sum_{j=1}^{m}{\bar{P}}_{i}\;;\;0\leq \lambda \leq 1,\;0\leq K_{i}\leq 1, \end{array}$$
 where $\lambda =\left(\sum_{i=1}^{m}{\bar{P}}_{i}|/|\sum_{i=1}^{m}{\bar{Q}}_{i}+\sum_{i=1}^{m}\bar{P}\right)$.
 Finally, alternatives can be ranked from the highest value of *K*_*i*_ to the lowest one.

## 3. Research Framework

The main purpose of the current study is to introduce a novel approach to identify and prioritize failure modes that result in MEs. In the first stage of this approach, the experts identify five factors that play an important role in MEs occurrence, including severity (*S*), occurrence (*O*), detection (*D*), cost (*C*), and time (*T*). The main reasons for the contribution of the aforementioned factors can be described as follows:

- *S*: identifying the severity of effects that patients will perceive in each failure mode
- *O*: understanding the likelihood of failure modes occur during the process
- *D*: detecting failure mode before the patient faces failure
- *C*: determining the amount of cost that can be wasted in each failure mode
- *T*: considering the urgency of time in each failure mode

Within the risk assessment range, the values of SODCT factors are defined using Table 6. Then, ten primary failure modes have been determined by the FMEA team through brainstorming (see Table 7). Afterward, the value of each risk factor for each failure mode is specified by experts. In this step, experts are asked to express the values of uncertainty and reliability using linguistic variables in order to use them in the following stages. In the second stage, the weights of risk factors are determined using the *Z*-SWARA method, introduced in Section 2.3, in an uncertain environment. In the third stage, the *Z*-WASPAS method, introduced in Section 2.4, is used to prioritize the identified failure modes with the aim of providing a distinct prioritization. To put it precisely, using the developed methods in the second and third stages can tackle some of the main disadvantages of the conventional FMEA technique, such as not assigning different weights to risk factors and not considering uncertainty and reliability in the process of determining the weight of factors and prioritizing failures. Finally, the results of the proposed approach are evaluated in comparison with conventional FMEA and fuzzy-WASPAS. A summary of the research framework has been presented in Figure 1.

## 4. Analysis of the Results

### 4.1. Proposed Approach Implementation

In this section, the results of implementing the proposed approach for assessing the influential failure modes in the MEs are presented. Initially, the value of each risk factor is determined by the FMEA team, and the results are presented in Table 8.

Then, according to FMEA team judgments, the values of SODCT factors for each failure mode are determined in the form of linguistic variables. These linguistic values of SODCT factors for ten identified failures are presented in Table 9.

In the second step of the proposed approach, for assigning weights to SODCT factors, the *Z*-SWARA method is used. For this purpose, first, experts in each group considered the most important criteria and then ordered other criteria in a descending form, from higher to lower importance, in comparison with the higher-ranked criteria. Thereafter, the order of each criterion is explained using linguistic variables and transformed into the form of *Z*-number based on Table 1 and Table 2. The results in the form of linguistic variables are indicated in Table 10. According to Table 5, these values are transformed to TFN, and then following the steps of *Z*-SWARA in Section 2.2, the weights of SODCT factors are calculated and summarized in Table 11.

To prioritize failure modes based on the *Z*-WASPAS method, initially, the decision-making matrix *H* of the *Z*-WASPAS method in the form of *Z*-numbers' components (considering reliability) was formed, where rows represent failure modes, and columns represent SODCT factors. Then, the decision-making matrix transforms into a matrix of TFN *H*, and consequently, ${\tilde{Q}}_{i}$ and ${\tilde{P}}_{i}$ are obtained. The results are shown in Table 12.

In Table 13, the average value of *Q*_*i*_and *P*_*i*_, the utility value *K*_*i*_, and the final rank of failure modes are presented. The value of *λ* is obtained equal to 0.48.

Based on Table 14, in the conventional FMEA method, F _5_ (entering patients ID numbers manually instead of scanning from bracelet) with RPN=8640 is at the top of the priority list to investigate in MEs occurrence. Furthermore, F _8_ (medication may be administered incorrectly via wrong route or dosage) is the second priority with RPN=8100, and F _3_ (mislabeling and incorrect medication dispensed in shelves in pharmacy) is the third with RPN=5670. The study of failures priority is indicated that based on conventional FMEA, ten failures have categorized into nine groups; the reason is the repetition of rank four in F _4_ (inability to verify the correctness of the given dose) and F _6_ (inappropriate ID scanning). This issue indicates that prioritizing, based on a traditional index, has not been perfectly done, and this issue results in the confusion of experts and decision-makers for planning corrective and preventive actions. Incomplete prioritizing of failure modes is the result of overlooking the weight of SODCT factors and uncertainty in ranking alternatives (see Table 14). In fuzzy-WASPAS and the proposed *Z*-WASPAS method, failure modes with greater *K*_*i*_ value are the main influential factors and rank in higher priorities. Utilizing the fuzzy-WASPAS method leads to improving the incomplete prioritizing problem of conventional FMEA in which the failure modes have been categorized into ten groups. Based on the fuzzy-WASPAS method, F _8_ (medication may be prepared wrongly via incorrect route or dosage) with *K*_*i*_=1.070, F _5_ with *K*_*i*_=1.046, and F _3_ with *K*_*i*_=1.020 are in first, second, and third priorities, respectively. Although the certainty is considered in weighting SODCT factors by the fuzzy-WASPAS method, the reliability has not contributed to the values of failure modes. Concerning the fact that reliability plays an important role in determining the most important failure modes in MEs, the proposed *Z*-WASPAS approach aims to synthesize the reliability of rating failure modes based on the expert's identification. In other words, including the reliability in the process of decision-making about significant failure modes can bring real results that are closer to reality and less injury to the patients. In the *Z*-WASPAS method, F _8_ with *K*_*i*_=1.01, F _5_ with *K*_*i*_=1.00, and F _3_ with *K*_*i*_=0.98 are in the first, second, and third priority, respectively.

### 4.2. Results Comparison

In this section, the outputs of the proposed approach have been compared with other similar methods to demonstrate its applicability. According to Table 14, in the fuzzy-WASPAS and *Z*-WASPAS method, the most significant failure mode is F _8_, whereas in the conventional FMEA, F _5_ is the most crucial failure mode. The main reason for this change is the nature of F _8_, in which there is considerable uncertainty about the wrong preparation of medication via incorrect route or dosage failure mode, among decision-makers (see Table 8). Assigning a weight to the SODCT factors and contributing uncertainty and unreliability in fuzzy-WASPAS and *Z*-WASPAS resulted in F _8_ being known as the main failure mode. The importance of *F*_8_ is the principal reason for this contradiction, which is determined by considering reliability. The importance of this failure mode was approved in several papers [56, 57]; any error occurrence in medication preparation can cause irreversible results for the patients or fatality.

F _3_ in all the methods ranks third place, which means that this failure mode has not been affected by weight changes, and the uncertainty is minimum about this failure mode based on experts' decision because of any mistake in stock of medication by the pharmacy can result in incorrect medication. The other failure modes affected by involving weight, uncertainty, and reliability and their ranks changed between four to ten.

The weight that is assigned to the S factor can have a considerable effect on the ranking since the severity plays an important role in MEs prevention. For instance, the fourth rank attributed to the F _4_ in conventional FMEA, but in fuzzy-WASPAS, the rank of this failure mode, one unit increased and stayed in the fifth rank. The main reason for this increment is the contributing weights of factors and certainty. However, when the reliability is involved in the ranking process, in the *Z*-WASPAS method, the ranking result for the F _4_ is the fourth alternative.  Figure 2 shows the comparisons of prioritizing failure modes according to three different methods.

One of the main problems that decision-makers face when using the conventional FMEA technique is assigning similar scores to different failure modes. In this case, decision-makers cannot properly identify critical failure modes and take corrective action to reduce their negative effects due to limited organizational resources. Therefore, this study tried to present the results with high separability compared to the FMEA by developing this conventional method based on the SWARA and WASPAS methods and using the *Z*-number theory. Besides, applying the concepts of uncertainty and reliability simultaneously in the *Z*-WASPAS method compared to the fuzzy-WASPAS can lead to more realistic results. In conclusion, based on FMEA methodology and the opinion of three experts (doctor, pharmacist, and nurse), F _5_ or manually entering the patient's ID and not scanning the patient bracelet is the principal reason of the MEs inducement, which would result in identifying the wrong ID or misuse of the medicine by the patient. However, in the proposed method, by involving reliability factors in identifying failure modes, F _8_ or medication administration error is known as a critical failure mode. Wu et al. [56] also confirmed the importance of this failure mode in MEs occurrence. The results also point to the importance of F _8_ as the main failure mode. The proposed corrective action is to ensure the information of the medicine, including dosage, route, and other administration specifics, that are immediately available in barcode medication administration. Moreover, F _5_ (entering patients identification numbers manually instead of scanning from bracelet) and F _3_ (incorrect medication dispensed in the drawer, or refrigerator, and mislabeling in pharmacy) were introduced as second and third main failure modes in MEs. Avoiding entering ID number unless approved by the charge nurse manually is the corrective action of F _5_ and having more than one pharmacy technician dispense medications at each section to double-check that medications are correctly dispensed is the corrective action for F _3_.

### 4.3. Sensitivity Analysis

A sensitivity analysis is administered by transforming the weight values of criteria in five different cases (see Table 15). Case _0_ represents the original crisp weights of the criteria that are obtained based on the *Z*-SWARA method in this research. For evaluating how the rank of alternatives changes in possible conditions, the crisp value of weights is assigned to the SODCT factors and made Case _1_ to Case _4_. The result of sensitivity analysis for ranking outcomes of ten failure modes and different cases is shown in Table 16. In this paper, the aggregated decision of three groups of decision-makers indicated that the order of importance in SODCT factors is *S*, *C*, *D*, *T*, and *O*, respectively. For instance, factor *S* has a significant impact on MEs' control in comparison with *C*. According to Table 16, F _8_ is the failure mode with the highest risk priority in all cases. Considering the SODCT factors, in Case _0_, Case _1_, and Case _3_, F _5_ is the second important failure mode because of the high weight of *S*, while in Case _2_ and Case _4_, F _3_ is the second significant failure mode because of the lower weight of *S*. This comparison is valid for other criteria and failure modes. The sensitivity analysis indicates that the weight of criteria can have a significant influence on the final ranking orders of failure modes. Therefore, determining the acceptable weight for criteria, according to the real situation, is of importance and advantage to the risk prioritization of failure modes and the subsequent corrective actions.

As stated, this study attempted to propose an extended approach using FMEA, SWARA, and WASPAS methods to prioritize MEs failure modes. In this approach, new factors of cost and time based on the case study in addition to traditional factors were added in comparison with the FMEA technique. Besides, this study tried to assign different weights to risk factors using the developed *Z*-SWARA method. This method has fewer pairwise comparisons compared to other conventional methods, such as the AHP method, and this research has considered the concepts of uncertainty and reliability in the process of determining the weights of risk factors simultaneously using the *Z*-SWARA method. In other methods like AHP or ANP, the model is created based on criteria and experts' evaluations that will affect priorities and ranks. So, SWARA can be useful for some issues whose priorities are known in advance according to situations [57]. Also, by developing the WASPAS method based on the *Z*-number theory and using it in the proposed approach, a more distinct prioritization of failures compared to the traditional RPN score has been presented.

## 5. Conclusion

One of the major causes of injury to patients when providing medical services is related to MEs. Identifying the MEs and reducing the likelihood of their occurrence is very important in order to increase the patient's level of safety. In this regard, using a decision-making approach based on the FMEA, a popular technique in this field, can help decision-makers identify and prioritize these errors. However, since this technique has some major drawbacks, this study has developed its proposed decision-making approach based on the *Z*-number theory. The proposed decision-making approach incorporates *Z*-SWARA and *Z*-WASPAS methods with the FMEA technique to address some disadvantages of the RPN score. In this research, by implementing and comparing the proposed approach with the conventional FMEA and fuzzy-WASPAS methods, the results indicated that prioritizing failure modes with the proposed method is closer to reality because of reliability factor involvement. On the other hand, the decision-makers can provide a series of appropriate corrective/preventive measures for critical failures, implement the corrective actions with the relevant departments, and perform a reassessment to examine the new situation and the effectiveness of these measures. Notably, failing to observe the cause-and-effect relation of failure modes is the main limitation of this study. Besides, not considering importance-necessity and uncertainty in decision making and addressing the relative importance among experts are the other issues that can be considered in future investigation using R-number, G-number, and evidence theories, respectively.

## Figures and Tables

**Figure 1:** Proposed research approach for prioritizing MEs failure modes.

**Figure 2:** Failure modes comparative ranking for the three different methods.

**Table 1:** Linguistic variables for weighting criteria [49].

Linguistic variables	TFNs
Equally important (EI)	(1, 1, 1)
Moderately less important (MOL)	(2/3, 1, 3/2)
Less important (LI)	(2/5, 1/2, 2/3)
Very less important (VLI)	(2/7, 1/3, 2/5)
Much less important (MUL)	(2/9, 1/4, 2/7)

**Table 2:** Linguistics variables for determining reliability [43].

Linguistic variables	Very weak (VW)	Weak (W)	Medium (M)	High (H)	Very high (VH)
TFNs	(0, 0, 0.25)	(0.2, 0.35, 0.5)	(0.35, 0.5, 0.75)	(0.5, 0.75, 0.9)	(0.75, 1, 1)

**Table 3:** Linguistic variables for rating failure modes [50].

Linguistic variables	Very poor (VP)	Poor (P)	Medium poor (MP)	Fair (F)	Medium good (MG)	Good (G)	Very good (G)
TFNs	(0, 1, 2)	(1, 2, 3)	(2, 3.5, 5)	(4, 5, 6)	(5, 6.5, 8)	(7, 8, 9)	(8, 9, 10)

**Table 4:** Transformation rules to convert *Z*-number to TFN $\left({\tilde{Z}}^{\prime }\right)$ based on linguistics variables for rating failure modes.

Linguistics variables	TFNs
(VP, VW)	(0, 0.29, 0.58)
(VP, W)	(0, 0.59, 1.18)
(VP, M)	(0, 0.73, 1.46)
(VP, H)	(0, 0.85, 1.69)
(VP, VH)	(0, 0.96, 1.91)
(P, VW)	(0.29, 0.58, 0.87)
(P, W)	(0.59, 1.18, 1.77)
(P, M)	(0.73, 1.46, 2.19)
(P, H)	(0.85, 1.69, 2.54)
(P, VH)	(0.96, 1.91, 2.87)
(MP, VW)	(0.58, 1.01, 1.44)
(MP, W)	(1.18, 2.07, 2.96)
(MP, M)	(1.46, 2.56, 3.65)
(MP, H)	(1.69, 2.96, 4.23)
(MP, VH)	(1.91, 3.35, 4.79)
(F, VW)	(1.15, 1.44, 1.73)
(F, W)	(2.37, 2.96, 3.55)
(F, M)	(2.92, 3.65, 4.38)
(F, H)	(3.39, 4.23, 5.08)
(F, VH)	(3.83, 4.79, 5.74)
(MG, VW)	(1.44, 1.88, 2.31)
(MG, W)	(2.96, 3.85, 4.73)
(MG, M)	(3.65, 4.75, 5.84)
(MG, H)	(4.23, 5.50, 6.77)
(MG, VH)	(4.79, 6.22, 7.66)
(G, VW)	(2.02, 2.31, 2.60)
(G, W)	(4.14, 4.73, 5.32)
(G, M)	(5.11, 5.84, 6.57)
(G, H)	(5.93, 6.77, 7.62)
(G, VH)	(6.70, 7.66, 8.62)
(VG, VW)	(2.31, 2.60, 2.89)
(VG, W)	(4.73, 5.32, 5.92)
(VG, M)	(5.84, 6.57, 7.30)
(VG, H)	(6.77, 7.62, 8.47)
(VG, VH)	(7.66, 8.62, 9.57)

**Table 5:** Transformation rules for *Z*-number to TFN based on linguistics variables for weighting criteria.

Linguistics variables	TFNs
(EI, VW)	(1, 1, 1)
(EI, W)	(1, 1, 1)
(EI, M)	(1, 1, 1)
(EI, H)	(1, 1, 1)
(EI, VH)	(1, 1, 1)
(MOL, VW)	(0.19, 0.29, 0.43)
(MOL, W)	(0.39, 0.59, 0.89)
(MOL, M)	(0.49, 0.73, 1.10)
(MOL, H)	(0.56, 0.85, 1.27)
(MOL, VH)	(0.64, 0.96, 1.44)
(LI, VW)	(0.12, 0.14, 0.19)
(LI, W)	(0.24, 0.30, 0.39)
(LI, M)	(0.29, 0.37, 0.49)
(LI, H)	(0.34, 0.42, 0.56)
(LI, VH)	(0.38, 0.48, 0.64)
(VLI, VW)	(0.08, 0.10, 0.12)
(VLI, W)	(0.17, 0.20, 0.24)
(VLI, M)	(0.21, 0.24, 0.29)
(VLI, H)	(0.24, 0.28, 0.34)
(VLI, VH)	(0.27, 0.32, 0.38)
(MUL, VW)	(0.06, 0.07, 0.08)
(MUL, W)	(0.13, 0.15, 0.17)
(MUL, M)	(0.16, 0.18, 0.21)
(MUL, H)	(0.19, 0.21, 0.24)
(MUL, VH)	(0.21, 0.24, 0.27)

**Table 6:** Traditional ratings for SODCT factors [55].

Rating	**S**	**O**	**D**	**C**	**T**
**10**	Hazardous with warning	Very high	Absolute	Repair cost close to the original price	Repair time extremely high
**9**	Hazardous without warning	Almost inevitable failure	Uncertainty	Repair cost extremely high	
**8**	Very high	High	High	Repair cost high	Repair time high
**7**	High	Repeated failures	Repeated failures		
**6**	Moderate	Moderate: occasional failures	Moderate: occasional failures	Repair cost moderately high	Repair time moderate
**5**	Low			Repair cost moderate	
**4**	Very low			Repair cost relatively low	
**3**	Minor	Low	Low	Repair cost low	Repair time low
**2**	Very minor	Relatively few failures	Relatively few failures	Repair cost very low	
**1**	None	Remote: failure is unlikely	Remote: failure is unlikely	Repair at nearly no cost	Repair cost very low

**Table 7:** Significant failure modes result in MEs.

Failure modes	Causes	Effects
Medication orders' confirmation		
F _1_: unable to verify medication orders	Absence of proper electronic health record (EHR).	Unable to know the dose that was given before.

Print medication list from electronic record		
F _2_: inaccessibility to EHR	Busy timetable, inappropriate communication.	Extra dose given.

Getting medication from pharmacy		

F _3_: mislabeling and incorrect medication dispensed in shelves in pharmacy	Misreading labels and incorrect stock of medications in pharmacy.	Giving incorrect medication, incorrect dose, or spending more time for giving the correct medication.
F _4_: unable to verify the correctness of given dose	Absence of supporting documentation to prove if patient received the dose before.	Incorrect medication administration.

Scan patient identification (ID) numbers		

F _5_: assigning incorrect ID number to patient	ID band is not scanned.	Medications might be administered to the wrong patient.
F _6_: inappropriate scanning	Busy timetable, lack of knowledge about medication administration.	Incorrect medication administration

Scan medication barcode and administrate		

F _7_: wrong medication or wrong time of administration process in pharmacy.	Mislabeling in pharmacy or physician changes the medication order.	Patient may not take the correct medication or receive medication at the right time.
F _8_: medication may be administered incorrectly via wrong route or dosage.	Wrongly reading order. Unfamiliarity with medicine.	The patient is negatively affected through incorrect route of medication.
F _9_: system overriding by manually entering medication barcode of medicines' containers.	Mislabeling of container. System malfunction.	Receiving the wrong medication, dose, or medication administration.

Prepare medications		

F _10_: medications may be prepared wrongly.	Incomprehensible medication label or physician order.	Patient may receive the incorrect dosage of medication or take the medication via the wrong route.
Incorrect dosage or incorrect route.	Not double-checking order previous to preparation.	

**Table 8:** Scoring risk factors based on FMEA team.

Failure mode	**S**			**O**			**D**			**C**			**T**		
	**TM**_**1**_	**TM**_**2**_	**TM**_**3**_	**TM**_**1**_	**TM**_**2**_	**TM**_**3**_	**TM**_**1**_	**TM**_**2**_	**TM**_**3**_	**TM**_**1**_	**TM**_**2**_	**TM**_**3**_	**TM**_**1**_	**TM**_**2**_	**TM**_**3**_
**F**_**1**_	3	4	5	4	5	5	1	1	2	5	3	4	4	3	5
**F**_**2**_	2	2	1	5	3	5	3	3	2	4	4	5	5	4	6
**F**_**3**_	8	7	5	3	3	4	9	7	6	9	8	9	4	5	6
**F**_**4**_	4	4	5	7	5	6	4	3	4	6	6	7	3	4	5
**F**_**5**_	8	8	9	5	6	5	8	9	10	6	4	6	4	3	5
**F**_**6**_	5	4	4	6	4	7	4	5	4	4	5	6	6	5	3
**F**_**7**_	2	2	3	4	2	3	10	8	10	3	2	4	5	3	4
**F**_**8**_	9	7	9	4	4	3	7	10	8	5	4	5	5	5	4
**F**_**9**_	8	7	8	4	3	4	5	8	7	4	4	5	3	4	2
**F**_**10**_	7	7	7	2	3	2	4	3	5	6	4	5	4	5	4

**Table 9:** The linguistic variable for the SODCT factors for each failure mode.

Risk factor	Teams	Failure modes									
		**F**_**1**_	**F**_**2**_	**F**_**3**_	**F**_**4**_	**F**_**5**_	**F**_**6**_	**F**_**7**_	**F**_**8**_	**F**_**9**_	**F**_**10**_
***S***	**TM**_**1**_	(ML, H)	(ML, M)	(H, VH)	(ML, M)	(EH, M)	(ML, VH)	(ML, VH)	(MH, H)	(H, M)	(MH, H)
	**TM**_**2**_	(M, M)	(L, VH)	(MH, M)	(MH, VH)	(H, H)	(M, M)	(L, H)	(H, M)	(MH, H)	(M, VH)
	**TM**_**3**_	(M, H)	(L, H)	(MH, M)	(M, M)	(H, M)	(M, VH)	(ML, M)	(VH, M)	(MH, M)	(MH, M)

***O***	**TM**_**1**_	(M, M)	(M, M)	(L, H)	(M, H)	(M, VH)	(M, H)	(L, M)	(M, H)	(ML, VH)	(L, H)
	**TM**_**2**_	(M, VH)	(MH, VH)	(ML, VH)	(M, VH)	(ML, H)	(MH, H)	(M, VH)	(ML, VH)	(ML, H)	(ML, H)
	**TM**_**3**_	(MH, M)	(MH, H)	(M, M)	(MH, H)	(MH, M)	(M, M)	(M, H)	(M, M)	(M, M)	(L, VH)

***D***	**TM**_**1**_	(L, H)	(M, M)	(MH, M)	(ML, H)	(MH, H)	(MH, M)	(H, H)	(MH, M)	(MH, VH)	(M, H)
	**TM**_**2**_	(L, VH)	(ML, H)	(H, M)	(ML, M)	(ML, VH)	(M, VH)	(H, M)	(H, VH)	(M, H)	(MH, VH)
	**TM**_**3**_	(ML, VH)	(L, H)	(H, VH)	(L, VH)	(MH, H)	(M, H)	(MH, VH)	(VH, H)	(MH, VH)	(M, H)

***C***	**TM**_**1**_	(M, H)	(ML, VH)	(MH, H)	(MH, H)	(M, H)	(ML, H)	(M, H)	(ML, H)	(M, M)	(ML, VH)
	**TM**_**2**_	(MH, M)	(ML, M)	(ML, M)	(MH, VH)	(MH, VH)	(ML, VH)	(M, H)	(M, H)	(MH, M)	(M, H)
	**TM**_**3**_	(M, M)	(M, M)	(M, H)	(M, H)	(M, H)	(ML, VH)	(ML, M)	(MH, M)	(M, M)	(ML, M)

***T***	**TM**_**1**_	(ML, H)	(M, H)	(MH, VH)	(ML, M)	(ML, M)	(M, H)	(ML, VH)	(M, H)	(L, H)	(ML, H)
	**TM**_**2**_	(M, VH)	(M, VH)	(M, H)	(M, M)	(ML, M)	(MH, VH)	(M-M)	(MH, VH)	(ML, M)	(ML, VH)
	**TM**_**3**_	(ML, H)	(M-H)	(MH-H)	(MH, VH)	(M-H)	(MH, VH)	(M-H)	(M-H)	(L-M)	(M-H)

**Table 10:** Prioritizing the SODCT factors based on their importance in TMs view.

TM_1_		TM_2_		TM_3_	
*S*		*S*		*C*	
***C***	(MOL, H)	***C***	(MOL, VH)	***S***	(VLI, M)
***O***	(VLI, H)	***T***	(LI, M)	***T***	(MOL, VH)
***T***	(MUL, M)	***D***	(VLI, H)	***O***	(LI, H)
***D***	(LI, VH)	***O***	(MUL, VH)	***D***	(MUL, H)

**Table 11:** Final weights of SODCT factors with *Z*-SWARA method.

Risk factor	**TM**_**1**_			**TM**_**2**_			**TM**_**3**_			Final weight		
	**a**	**B**	**c**	**a**	**b**	**C**	**a**	**B**	**c**	**a**	**b**	**c**
***S***	0.329	0.362	0.404	0.359	0.412	0.484	0.152	0.211	0.289	0.280	0.328	0.392
***C***	0.257	0.293	0.336	0.148	0.211	0.296	0.342	0.388	0.450	0.249	0.297	0.361
***O***	0.106	0.151	0.205	0.059	0.099	0.153	0.094	0.141	0.201	0.086	0.130	0.187
***T***	0.068	0.106	0.154	0.100	0.156	0.230	0.114	0.165	0.232	0.094	0.143	0.205
***D***	0.055	0.088	0.130	0.075	0.122	0.185	0.058	0.095	0.146	0.062	0.102	0.154

**Table 12:** Aggregated weighted normalized decision matrix of WSM (WPN).

Failure modes	***S***			***O***			***D***			***C***			**T**		
	**a**	**b**	**c**	**A**	**b**	**c**	**A**	**b**	**c**	**a**	**b**	**C**	**a**	**b**	**C**
**F**_**1**_	0.08 (0.62)	0.17 (0.80)	0.32 (0.98)	0.05 (0.87)	0.11 (0.97)	0.22 (1.07)	0 (0.71)	0.02 (0.85)	0.06 (0.94)	0.11 (0.74)	0.23 (0.92	0.45 (1.13)	0.03 (0.79)	0.08 (0.92)	0.18 (1.03)
**F**_**2**_	0.01 (0.32)	0.06 (0.58)	0.19 (0.83)	0.07 (0.92)	0.13 (1.0)	0.25 (1.1)	0.01 (0.8)	0.03 (0.88)	0.07 (0.96)	0.05 (0.59)	0.15 (0.81)	0.35 (1.04)	0.05 (0.85)	0.11 (0.96)	0.22 (1.065)
**F**_**3**_	0.2 (0.85)	0.3 (0.97)	0.47 (1.12)	0.02 (0.77)	0.06 (0.9)	0.15 (1)	0.07 (0.95)	0.07 (0.99)	0.14 (1.03)	0.1 (0.72)	0.220.91	0.45 (1.13)	0.07 (0.9)	0.14 (0.99)	0.27 (1.09)
**F**_**4**_	0.11 (0.7)	0.2 (0.85)	0.36 (1.03)	0.06 (0.9)	0.12 (0.99)	0.24 (1.08)	0.01 (0.75)	0.03 (0.86)	0.06 (0.95)	0.16 (0.82)	0.3 (1.0)	0.58 (1.22)	0.05 (0.85)	0.1 (0.95)	0.21 (1.05)
**F**_**5**_	0.23 (0.89)	0.33 (1.0)	0.48 (1.13)	0.05 (0.87)	0.1 (0.96)	0.21 (1.6)	0.04 (0.9)	0.07 (0.96)	0.12 (1.01)	0.13 (0.78)	0.27 (0.97)	0.53 (1.19)	0.02 (0.77)	0.07 (0.90)	0.16 (1.01)
**F**_**6**_	0.09 (0.64)	0.18 (0.82)	0.34 (1.01)	0.06 (0.89)	0.11 (0.98)	0.22 (1.07)	0.04 (0.9)	0.07 (0.95)	0.11 (1.0)	0.04 (0.53)	0.15 (0.81)	0.36 (1.05)	0.08 (0.91)	0.15 (1.0)	0.28 (1.1)
**F**_**7**_	0.02 (0.42)	0.1 (0.66)	0.23 (0.88)	0.03 (0.83)	0.08 (0.93)	0.18 (1.04)	0.07 (0.95)	0.1 (0.99)	0.14 (1.03)	0.08 (0.67)	0.19 (0.87)	0.4 (1.09)	0.04 (0.81)	0.09 (0.93)	0.19 (1.04)
**F**_**8**_	0.23 (0.88)	0.32 (0.98)	0.46 (1.11)	0.04 (0.84)	0.09 (0.95	0.19 (1.05)	0.08 (0.97)	0.11 (1.0)	0.14 (1.03)	0.09 (0.70)	0.21 (0.90)	0.43 (1.11)	0.06 (0.88)	0.13 (0.98)	0.25 (1.08)
**F**_**9**_	0.19 (0.83)	0.28 (0.95)	0.44 (1.10)	0.02 (0.80)	0.07 (0.92	0.17 (1.03)	0.05 (0.93)	0.08 (0.98)	0.14 (1.03)	0.11 (0.73)	0.22 (0.90)	0.43 (1.11)	0 (0.6)	0.031 (0.79)	0.1 (0.94)
**F**_**10**_	0.16 (0.78)	0.26 (0.92)	0.43 (1.09)	0 (0.65)	0.04 (0.84)	0.12 (0.98)	0.04 (0.91)	0.07 (0.96)	0.12 (1.01)	0.06 (0.61)	0.17 (0.83)	0.37 (1.07)	0.03 (0.78)	0.08 (0.92)	0.18 (1.03)

**Table 13:** Final result of ranking failure modes for *λ* = 0.48

Failure modes	**Q** _**i**_	**P** _**i**_	**K** _**i**_	Rank
**F**_**1**_	0.709	0.648	0.677	8
**F**_**2**_	0.593	0.492	0.541	10
**F**_**3**_	0.918	0.874	0.895	3
**F**_**4**_	0.866	0.788	0.825	4
**F**_**5**_	0.942	0.893	0.917	2
**F**_**6**_	0.760	0.710	0.734	5
**F**_**7**_	0.647	0.583	0.614	9
**F**_**8**_	0.941	0.904	0.922	1
**F**_**9**_	0.781	0.703	0.740	6
**F**_**10**_	0.710	0.659	0.683	7

**Table 14:** Failure modes prioritization using the proposed approach compared to other methods.

Failure modes	Conventional FMEA		Fuzzy-WASPAS		*Z*-WASPAS	
	RPN	Rank	**K**_**i**_	Rank	**K**_**i**_	Rank
**F**_**1**_	800	8	0.791	6	0.74	8
**F**_**2**_	600	9	0.605	10	0.60	10
**F**_**3**_	5670	3	1.020	3	0.98	3
**F**_**4**_	3600	4	0.908	5	0.91	4
**F**_**5**_	8640	1	1.046	2	1.00	2
**F**_**6**_	3600	4	0.764	7	0.81	5
**F**_**7**_	1215	6	0.685	9	0.68	9
**F**_**8**_	8100	2	1.070	1	1.01	1
**F**_**9**_	3360	5	0.917	4	0.81	6
**F**_**10**_	1120	7	0.758	8	0.75	7

**Table 15:** Weights and crisp value of weights of SODCT factors in different cases.

Risk factor	Case _0_	Case _1_	Case _2_	Case _3_	Case _4_
**w**_**S**_	(0.28, 0.33, 0.39)	(0.26, 0.30, 0.35)	(0.22, 0.33, 0.29)	(0.53, 0.38, 0.48)	(0.02, 0.12, 0.09)
*α*_**w**_**S**__	0.333	0.3	0.28	0.46	0.08
**w**_**O**_	(0.09, 0.13, 0.19)	(0.09, 0.06, 0.14)	(0.02, 0.05, 0.09)	(0.02, 0.01, 0.03)	(0.20.12, 0.26)
*α*_**w**_**O**__	0.134	0.1	0.05	0.02	0.19
**w**_**D**_	(0.06, 0.10, 0.15)	(0.26, 0.15, 0.35)	(0.29, 0.23, 0.32)	(0.12, 0.08, 0.14)	(0.35, 0.25, 0.28)
*α*_**w**_**D**__	0.106	0.25	0.28	0.11	0.29
**w**_**C**_	(0.25, 0.30, 0.36)	(0.29, 0.23, 0.39)	(0.15, 0.01, 0.17)	(0.39, 0.20, 0.29)	(0.25, 0.32, 0.29)
*α*_**w**_**C**__	0.302	0.3	0.11	0.29	0.29
**w**_**T**_	(0.09, 0.14, 0.21)	(0.02, 0.08, 0.05)	(0.22, 0.29, 0.32)	(0.10, 0.09, 0.18)	(0.20, 0.09, 0.15)
*α*_**w**_**T**__	0.147	0.05	0.28	0.12	0.15

**Table 16:** Ranking results of failure modes with respect to the different cases.

Failure modes	Case _0_	Case _1_	Case _2_	Case _3_	Case _4_
**F**_**1**_	8	9	9	8	9
**F**_**2**_	10	10	10	10	10
**F**_**3**_	3	3	2	3	2
**F**_**4**_	4	5	8	5	6
**F**_**5**_	2	2	3	2	3
**F**_**6**_	5	7	4	7	4
**F**_**7**_	9	8	7	9	5
**F**_**8**_	1	1	1	1	1
**F**_**9**_	6	4	6	4	7
**F**_**10**_	7	6	5	6	8

## Data Availability

The data are extracted by experts sorting criteria, from the most important to less important in descending order, based on self-identification.
